# Intervention Effect of Group Counseling Based on Positive Psychology on Psychological Crisis of College Student

This article has been retracted.

**DOI:** 10.1155/2022/3132016

**Published:** 2022-08-12

**Authors:** Zixi Zhang, Yabo Li, Sailan Sun, Ziye Tang

**Affiliations:** ^1^Qiannan Normal College for Nationalities, Duyun, China; ^2^Qiannan Nationality Professional Technology College, Qiannan, China

## Abstract

**Objective:**

To analyze the intervention effect of group counseling based on positive psychology on psychological crisis of college student.

**Method:**

SCL-90 mental health screening was performed on second-year students in a college by cluster stratification. Among the detected students, 210 were included into the group after brief interview and randomly assigned to the experimental group and the control group. The control group was given conventional intervention measures, and the experimental group was given group counseling according to the interview results. One week before the start, on the day of the end of the intervention and 3 months after the end of the intervention, the mental health level of all subjects was evaluated by symptom self-rating scale, general well-being scale, and adolescent mental resilience scale.

**Results:**

The scores of two groups were different at different time points during the intervention. With the extension of time, the score of the self-rating symptom scale in the experimental group decreased significantly, while the total score of the self-rating symptom scale in the control group increased, with statistical significance (*P* < 0.05). Before the intervention, there was no significant difference in general well-being between the two groups (*P* > 0.05). At 3 months after the end of intervention, the total score of the general well-being scale in the experimental group increased, while that in the control group decreased, with statistical significance (*P* < 0.05). Three months after the end of the intervention, the total score of adolescent mental resilience scale in the experimental group increased.

**Conclusion:**

Group counseling from the perspective of positive psychology can effectively improve the mental health status of medical students with psychological crisis and improve their mental resilience.

## 1. Introduction

Due to the influence of different cultures and family backgrounds, some college students cannot well adapt to the current campus life and interpersonal environment, and there are various psychological and interpersonal barriers. With the help of group psychological counseling to intervene students' mental health, it promotes students to better integrate into group activities, campus environment, and social environment [1]. In recent years, the trend of positive psychology led by the famous American psychologist, Martin Seligman, has gradually entered the field of vision of researchers [2]. Its value orientation is to focus on mental illness, instead of focusing on the good beings to assist people explore and inspire their inner qualities and strength, and achieve a better life [3, 4]. Compared with psychology, positive psychology emphasizes solving people's psychological problems with a more positive mentality and ideas. With the help of this positive and optimistic psychology, people are more willing to open their hearts and tell their problems [5]. At present, the empirical research with positive psychology theory as the core, especially the absolute number of group counseling, is still relatively small. There are few studies on the general intervention of psychological crisis, which mainly focus on poor students and depression [6]. Students entering colleges are faced with great changes in living environment, learning style, and interpersonal relationship [7]. For college students' health educators, it is to make college students aware of their positive quality with the help of scientific measurement methods, strengthen their positive personality through active intervention, and then form a healthy psychology [8]. However, the psychological development is relatively backward, which will inevitably bring them great pressure and psychological confusion to adapt and develop, and it is easy to produce psychological crisis [9]. Crisis intervention is to give care and support to the people who are in trouble or suffer setbacks so as to restore their psychological balance [10, 11]. With the help of the original psychological related scales such as the symptom self-rating scale (SCL-90), general well-being scale (GWB), and adolescent mental resilience scale (KHRA), many colleges and universities have also compiled psychological related scales to scientifically obtain the psychological dynamics and related indicators of college students and obtain data sources for better providing psychological services for students [12–14].

In this study, SCL-90 mental health screening was performed on second-year students in a college by cluster stratification. Among the detected students, 210 were included into the group after brief interview. The experimental group was given group counseling according to the interview results. The positive psychology-oriented group counseling method was adopted to intervene the psychological crisis group of students in a college. The contribution of this study can not only provide an opportunity for college students to grow up in mental health but also provide a reference for the improvement of college students' psychological crisis intervention model. The chapter arrangement of this study is shown in Figure 1.

## 2. Materials

### 2.1. Basic Materials

A total of 210 students effectively participated in the whole intervention, including 105 in the experimental group, 43 males and 62 females, aged (20.38 ± 1.21) years old. 47 males and 58 females in control group, aged (20.44 ± 0.73) years. The relevant information of students is shown in Table 1.

### 2.2. Inclusion Criteria

① The UPI scale was selected as the first category [15], which was the total score and was greater than 25 points; the answer to the 25 question “want to take a life” was affirmative; there were more than two auxiliary questions for the affirmative; the consulting requirements were clearly put forward
② With negative emotions, behavior, and physical changes
③ Volunteered to participate in the study

### 2.3. Exclusion Criteria

① Had been diagnosed with severe depression, neurosis, and schizophrenia
② Other unsuitable candidates

## 3. Methodology

### 3.1. Grouping Method

With the support of school and psychological teachers, the second-year students of a college by cluster stratification for mental health screening were selected. In accordance with the principle of voluntary recruitment, 210 students were included into the group after a brief interview. Students were asked to fill in three scales: the symptom self-rating scale (SCL-90), general well-being scale (GWB), and adolescent mental resilience scale (KHRA) to obtain the data needed for the research.

### 3.2. Control Group

The control group took the conventional intervention measures and participated in the psychological health lecture conducted by the school, once a week, in the form of large class in the amphitheater. The school sets up a psychological counseling office; colleges and departments are equipped with full-time psychological counseling teachers; psychological publicity materials were distributed to students every academic year; students were organized to listen to educational lectures in case of valuable cases.

### 3.3. Experimental Group

The experimental group set the intervention plan according to the interview results and carried out group counseling with positive psychology concept as the core. The subjects in the experimental group were divided into 4 groups with 26 ∼ 27 members in each group. The researcher himself was the group leader. The counseling program was based on the concept of positive psychotherapy and applied research as the core, combined with theoretical lectures and practical activities and other forms of design, focusing on positive cognition, emotional training, and practical problem solving.

1. In the aspect of cultivating positive cognition, the students' perception was touched mainly through theory introduction, role play, self-confidence training, and summary after the activity. The main areas are as follows: ① external signs, ② inner spiritual world, and ③ their position in the collective.
2. In terms of cultivating positive emotions, students should create a positive and joyful atmosphere through warm-up activities, relaxation meditation, and other methods [16]. Students can also take the following ways to cultivate positive emotions: ① appreciate others as much as possible, ② do not always compare yourself with others, ③ self-guidance, ④ act in an optimistic way, ⑤ live now, and ⑥ make more mental preparations before doing things.
3. In terms of solving practical problems, students should clarify the truth with the help of games or stories and guide students to apply it by arranging tasks or reproducing cases. At the same time, students were encouraged to expose their own problems and get support and help from their peers in the group. To improve the effectiveness of group coaching, participants were asked to keep a diary of their daily positive perceptions, experiences, or related events during the study period. The total intervention time was 6 weeks, once a week, about 2.5 h each time. The researchers were qualified as psychological counselors and had received relevant group training.

### 3.4. Observational Index

One week before the start of the intervention, all the subjects were assessed for their mental health with the symptom self-rating scale, general well-being scale, and adolescent mental resilience scale. The recovery rate and effective rate of the questionnaire were 100%. The assessment at the end of the intervention reflected the immediate effect of the intervention, and the assessment at 3 months after the end of the intervention reflected the short-term maintenance effect of the intervention.

1. The symptom self-rating scale (SCL-90) [17]: SCL-90 is one of the commonly used mental health test scales in the world and it will help you understand your mental health from ten aspects. This test is applicable to people over 16 years old. There were 90 rating items on a scale of 1 to 5.
2. General well-being scale (GWB) [18]: GWB is a customized test tool developed for the National Center for health statistics to evaluate subjects' statements of happiness, in the first 18 of 33 items in this study.
3. Adolescent mental resilience scale (KHRA) [19]: the adolescent mental resilience scale (KHRA) was developed by psychologists in California based on the dynamic model of resilience. There were 27 items, all of which were rated from 1 to 5, with high scores and good mental toughness.

### 3.5. Statistical Methods

SPSS 24.0 software was used for data analysis. Two independent samples *t*-test was used for comparison between groups. *P* < 0.05 indicated a statistically significant difference.

## 4. Results

### 4.1. Result of Symptom Self-Rating Scale

With the extension of time, the score of the self-rating symptom scale in the experimental group decreased significantly, while the total score of the self-rating symptom scale in the control group increased, with statistical significance (*P* < 0.05). Result of symptom self-rating scale is shown in Table 2.

### 4.2. Result of General Well-Being Scale

At 3 months after the end of intervention, the total score of the general well-being scale in the experimental group increased, while that in the control group decreased, with statistical significance (*P* < 0.05). Result of general well-being scale is shown in Table 3.

### 4.3. Result of Adolescent Mental Resilience Scale

The results of adolescent resilience between the two groups (*P* > 0.05). Three months after the end of the intervention, the total score of adolescent mental resilience scale in the experimental group increased, which was statistically significant (*P* < 0.05). Result of adolescent mental resilience scale is shown in Table 4.

## 5. Discussion

Positive psychology advocates to cultivate positive psychological qualities, stimulate positive potential, help individuals maintain the balance and stability of psychological state, improve mental toughness, and prevent the occurrence and progress of psychological crisis of students [6, 20]. Schools do not pay enough attention to students' mental health education, which leads to the imperfect mechanism of mental health education. Schools should actively adjust the way of psychological work, rely on the research theory of positive psychology, and effectively improve the content and way of psychological work education [21, 22]. The students in colleges are in the transition stage from “school people” to “social people.” The psychology is not mature enough and is easy to fall into a state of psychological crisis. However, in addition to the potential self-psychological conflict, students in psychological crisis also have internal self-improvement ability [23]. The essence of positive psychological intervention is to make students realize that external or internal dilemmas may be inevitable, but they can explore their own advantages [24]. Schools put forward the mental health education strategies of paying attention to the positive level of psychology, actively facing psychological problems, active prevention, and active and effective intervention, which solve the psychological problems of special college students [25]^.^Group counseling provides a platform for students to accept and practice the thoughts of positive psychology through general comfort function, reference reflection function, forerunner example function, test field feedback function, and other group interaction mechanism [26]. Positive psychology-oriented intervention is to develop, cultivate, and guide this potential, while group counseling makes it possible to practice the concept of positive change [27]. Positive psychology can promote individual subjective well-being, and it is especially suitable for mental health education in colleges and universities. Group counseling is a form of psychological counseling by creating group situation and using group dynamics, and it is one of the effective ways to implement college students' mental health education, adjust their relationship with others, and learn new ways of behavior [28]. Life meaning group counseling can improve the psychological symptoms of college freshmen [29]. Compared with individual intervention, it is a feasible way to maintain the mental health of students in colleges [30].

Research in this study showed that the scores were different at different time points during the intervention. With the extension of time, the score of the self-rating symptom scale in the experimental group decreased significantly, while the total score of the self-rating symptom scale in the control group increased, with statistical significance (*P* < 0.05). Before the intervention, there was no significant difference in general well-being between the two groups (*P* > 0.05)). At 3 months, after the end of intervention, the total score of the general well-being scale in the experimental group increased, while that in the control group decreased, with statistical significance (*P* < 0.05). Before the intervention, there was no significant difference in the results of adolescent resilience between the two groups (*P* > 0.05)). Three months after the end of the intervention, the total score of adolescent mental resilience scale in the experimental group increased.

## 6. Conclusion

In conclusion, group counseling from the perspective of positive psychology can effectively improve the mental health status of students with psychological crisis and improve their mental resilience; it can also help students develop easygoing, confident, optimistic, positive, sharp, and careful character, as well as their strong field control ability and adaptability; it provides a reference for the improvement of college students' psychological crisis intervention model. The integrity of the results obtained in this study may not be high. We hope that future scholars can collect a large sample size and study the mental health status of college students in many ways in combination with off-campus group activities, skill competitions, quality development, and other activities.

## Figures and Tables

**Figure 1:** The chapter arrangement of this study.

**Table 1:** General information of cases.

Groups	Cases	Average age
Experimental group	43 males	20.38 ± 1.21
	62 females	

Control group	47 males	20.44 ± 0.73
	58 females	

**Table 2:** Result of symptom self-rating scale (SCL-90).

Groups	*n*	Before intervention	End of intervention	3 months after intervention	*F* (time effect)	*F* (interaction effect)
Experimental group	105	179.65 ± 19.64	154.38 ± 24.65	154.05 ± 20.36	19.676	15.449
Control group	105	176.58 ± 23.44	172.47 ± 32.26	177.56 ± 24.17		
*t*		0.568	2.581	4.338		
*P*		>0.05	<0.05	<0.05		

**Table 3:** Result of general well-being scale (GWB).

Groups	*n*	Before intervention	End of intervention	3 months after intervention	*F* (time effect)	*F* (interaction effect)
Experimental group	105	72.85 ± 8.14	77.62 ± 8.31	78.09 ± 8.82	2.805	5.236
Control group	105	71.72 ± 11.13	72.27 ± 12.13	69.58 ± 7.16		
*T*		0.501	2.120	4.283		
*P*		>0.05	<0.05	<0.05		

**Table 4:** Result of adolescent mental resilience scale (KHRA).

Groups	*n*	Before intervention	End of intervention	3 months after intervention	*F* (time effect)	*F* (interaction effect)
Experimental group	105	93.46 ± 8.34	99.72 ± 7.32	99.86 ± 6.78	2.345	15.318
Control group	105	96.41 ± 10.22	94.62 ± 10.01	92.54 ± 8.23		
*T*		1.391	2.337	3.875		
*P*		>0.05	<0.05	<0.05		

## Data Availability

The data used to support the findings of this study are included within the article.

## References

[1] Gao L., Huang G., Yan J., Li H. (2022). Research on the influence of group psychological counseling on mental health intervention of poor college students the Yellow River Loess. *Yellow people*.

[2] Choi Y. H., Kim J. H. (2015). The study of mid-life crisis using positive psychology. *Korean Review of Management Consulting*.

[3] Kim J. E. (2016). The effects of positive psychology-based group counseling program on positivity and school adjustment resilience of school violence perpetrators. *Journal of Social Sciences*.

[4] Javid N., Ahmadi A., Mirzaei M., Atghaei M. (2019). Effectiveness of solution-focused group counseling on the mental health of midwifery students. *Revista Brasileira de Ginecologia e Obstetrícia/RBGO Gynecology and Obstetrics*.

[5] Zou H. (2019). The concept and development trend of positive psychology. *Management observation*.

[6] Flynn C., Sharma M. M. (2016). Mental health aspects of responding to campus crises. *New Directions for Student Services*.

[7] Wang Z. (2018). College students coping with psychological crisis from the perspective of health management [J]. *Journal of Shenyang Institute of Education*.

[8] Dang Z. (2020). Development strategy of College Students’ mental health based on positive psychology. *[J] Encyclopedia knowledge*.

[9] Bitsios P., Karademas E., Mouzaki A. (2017). The student counselling centre at the university of crete, Greece. *BJPsych International*.

[10] Gazda G., Ohlsen M. (2014). The Effects of short-term group counseling on prospective counselors [J]. *Journal of Counseling and Development*.

[11] Liu M., Cao G., Sun Z. (2019). Study on the intervention of college students’ psychological crisis grades [J]. *Chinese Journal of Health Emergency Electronic*.

[12] He hang, Bao W. (2021). The impact of the COVID-19 on the mental health of College Students -- Taking the SCL-90 psychological assessment of sophomores in a university as an example. *[J] Intelligence*.

[13] Li D. (2008). *Compilation of Mental Health Scale for College Students [D]*.

[14] Xu C. (2013). Compilation of College Students’ sexual and mental health scale -- Based on the mathematical statistical analysis of the survey data of six schools in Jinan. *[J] China Science and education innovation guide*.

[15] Deng C., Wang L. (2018). A comparative study of UPI and SCL-90 assessment results for freshmen in private colleges [J]. *Statistics and Management*.

[16] Currier J. M., Deiss J., Mcdermott R. C. (2017). From whom do student veterans seek help?: understanding the roles of professional, informal, and religious sources [J]. *The Journal of Nervous and Mental Disease*.

[17] Yang L. (2019). Comparison of symptom self-rating scale and college students personality questionnaire on mental health status in higher vocational colleges [J]. *Modern Vocational Education*.

[18] Alagheband M., Ahmadabadi N. M., Abdollahi A. S. (2013). Psychometric characteristics of the general well-being schedule (GWB) in an Iranian sample [J]. *Life Science Journal*.

[19] Liu Q., Wang M., Xiang Q. (2016). The relationship between adolescent resilience and parenting style [J]. *Chinese Journal of Health Psychology*.

[20] Olekalns M., Horan C. J., Smith P. L. (2014). Maybe it’s right, maybe it’s wrong: structural and social determinants of deception in negotiation. *Journal of Business Ethics*.

[21] Pan Y., Yin T., Wu L. (2022). On the working mechanism of mental health education in Colleges and universities from the perspective of positive psychology. *[J] Psychological monthly*.

[22] Chen Q. (2021). Research on the full membership and long-term mechanism of College Students’ mental health education from the perspective of positive psychology. *[J] University*.

[23] Nakimuli-Mpungu E., Okello J., Kinyanda E. (2013). The impact of group counseling on depression, post-traumatic stress and function outcomes: a prospective comparison study in the Peter C. Alderman trauma clinics in northern Uganda. *Journal of Affective Disorders*.

[24] Kivlighan D. M., Tibbits B. M. (2012). Silence is mean and other misconceptions of group counseling trainees: identifying errors of commission and omission in trainees’ knowledge structures. *Group Dynamics: Theory, Research, and Practice*.

[25] Fu X. (2012). Application of group psychological counseling in college student management. *[J] Jiangsu higher education*.

[26] Wang X. (2018). Study on prevention and intervention of psychological crisis of college students in higher vocational colleges [J]. *Journal of Lianyungang Vocational and Technical College*.

[27] ÜzarÖzçetin Y. S., Hiçdurmaz D. (2017). Effects of structured group counseling on anger management skills of nursing students. *Journal of Nursing Education*.

[28] Lee M. H., Kim J. (2018). The effect of adlerian group counseling program on responses to inferiority feelings among university students. *Korean Journal of Youth Studies*.

[29] Liu H., Yang Y., Wang W., Zhao R., Chen X., Yang J. (2020). Effect of life meaning group counseling on psychological symptoms of college freshmen. *[J] Chinese Journal of mental health*.

[30] Li Y. (2019). Study on the intervention effect of hope trait group counseling on college students’ test anxiety [J]. *Chinese Journal of Clinical Psychology*.

